# “Not for All the Tea in China!” Political Ideology and the Avoidance of Dissonance-Arousing Situations

**DOI:** 10.1371/journal.pone.0059837

**Published:** 2013-04-19

**Authors:** H. Hannah Nam, John T. Jost, Jay J. Van Bavel

**Affiliations:** Department of Psychology, New York University, New York, New York, United States of America; Ecole Normale Supérieure, France

## Abstract

People often avoid information and situations that have the potential to contradict previously held beliefs and attitudes (i.e., situations that arouse cognitive dissonance). According to the motivated social cognition model of political ideology, conservatives tend to have stronger epistemic needs to attain certainty and closure than liberals. This implies that there may be differences in how liberals and conservatives respond to dissonance-arousing situations. In two experiments, we investigated the possibility that conservatives would be more strongly motivated to avoid dissonance-arousing tasks than liberals. Indeed, U.S. residents who preferred more conservative presidents (George W. Bush and Ronald Reagan) complied less than Americans who preferred more liberal presidents (Barack Obama and Bill Clinton) with the request to write a counter-attitudinal essay about who made a “better president.” This difference was not observed under circumstances of low perceived choice or when the topic of the counter-attitudinal essay was non-political (i.e., when it pertained to computer or beverage preferences). The results of these experiments provide initial evidence of ideological differences in dissonance avoidance. Future work would do well to determine whether such differences are specific to political issues or topics that are personally important. Implications for political behavior are discussed.

## Introduction

*I know that most men…can very seldom discern even the simplest and most obvious truth if it be such as to oblige them to admit the falsity of conclusions they have formed, perhaps with much difficulty – conclusions of which they are proud, which they have taught to others, and on which they have built their lives.* (Leo Tolstoy [1]).

In some sense, the fulfillment of democratic ideals depends upon the capacity and motivation of citizens to be active, attentive participants in civil discourse and to be capable of processing political information objectively. Unfortunately, the consensus among political scientists is that “citizens [are] on average subpar with respect to what is required by classical democratic theory on almost every dimension” [2], [3]. Evidence of biased, motivated reasoning in the political domain is easy to find [4], [5], [6], [7]. At the same time, some citizens seem to be more logical, thoughtful, and open-minded than others [8], [9], [10]. Some evidence suggests, albeit tentatively, that ideological asymmetries may exist when it comes to the role of motivation in political reasoning as practiced by liberals and conservatives [11], [12], [13], [14], [15], [16].

### Political Ideology as Motivated Social Cognition

Even a cursory analysis of the political landscape in the contemporary United States reveals that there are vast differences in the cognitive and rhetorical styles of liberals and conservatives – as reflected, say, in the differences between National Public Radio and Fox News or Jon Stewart and Rush Limbaugh. Increasingly, ideological polarization is the norm, and little or no common ground exists between liberals and conservatives when it comes to social and economic issues such as tax policy, the debt ceiling, health care reform, gay marriage, and climate change [17], [18], [19]. Undoubtedly, ideological conflict is fostered (at least in part) by institutional, system-level processes, such as electoral competition between political parties and the organized activities of lobbyists. At the same time, there is growing evidence that differences between liberals and conservatives are shaped by psychological variables having to do with personality, cognition, emotion, and motivation – all of which may help to explain why the preferences and styles of liberals and conservatives often diverge [20].

In seeking to integrate social psychological theories of motivated social cognition with historical and philosophical accounts of political ideology, Jost, Glaser, Kruglanski, and Sulloway [21] proposed that situational and dispositional variability in basic orientations toward uncertainty and threat help to explain why conservatives are more resistant to change and more accepting of inequality, in comparison with liberals. They conducted a meta-analytic review of the available evidence and concluded that, among other things, conservatives possess stronger needs for order, structure, consistency, and closure and weaker tolerance for ambiguity and threat than liberals. Subsequent research in psychology and neuroscience has corroborated the notion that, all other things being equal, adherence to conservative (vs. liberal) ideology is associated with certainty-oriented forms of epistemic motivation and behavior, including inhibition-based avoidance (vs. approach) motivation as well as cognitive rigidity [22]; persistence in dominant or habitual response patterns in the face of conflicting task requirements that require flexibility [23]; the pursuit of cautious, less exploratory learning strategies [24]; and a reluctance to acknowledge and engage in integrative policy trade-offs involving potentially conflicting values [25]. These and other findings are suggestive of the intriguing possibility that conservatives would respond more negatively than liberals to situations that arouse cognitive dissonance.

### Cognitive Dissonance Theory

According to Festinger's [26] cognitive dissonance theory, psychological tension (or dissonance) arises whenever an individual simultaneously holds two or more fundamentally conflicting cognitions, such as (a) I like to smoke cigarettes, and (b) the scientific evidence indicates that tobacco smoking causes cancer and many other serious health problems. The dissonance leads individuals to try to reduce inconsistency one way or another – such as by quitting smoking, disparaging the scientific evidence, or concluding that long life is overrated [27]. Festinger [26] suggested that people are motivated to avoid even *considering* information that is inconsistent with their preexisting views and preferences, insofar as such information will be inherently dissonance-arousing.

Over the years, a great number of studies have identified *selective exposure* as a proactive strategy for minimizing cognitive dissonance [14]. In one of the earliest demonstrations, Hyman and Sheatsley [28] observed that people tend to seek out information that is compatible with their preexisting beliefs and to avoid exposure to information that is incompatible with their preexisting beliefs and opinions. The phenomenon of selective exposure has been observed in a variety of consequential decision-making domains. Examples include smokers' evasion of information that spells out the connection between smoking and cancer [29], medical patients' preferences for ignorance concerning severe health risks [30], and selective inattention to attitude-incongruent data on the part of ideological opponents of affirmative action and gun control [7].

Although motivated avoidance of unwelcome or contradictory information is quite common, there are cross-cultural and inter-individual differences in the ways in which people respond to dissonance-arousing situations [31], [32], [33] and engage in selective exposure [34]. Individuals who are dispositionally high (vs. low) in the need for consistency are especially likely to report psychological discomfort in response to conflicting cognitions [35]. In addition, it appears that threat causes individuals who are high in authoritarianism to exhibit an even stronger preference for exposure to one-sided, pro-attitudinal information [36]. Low authoritarians, by contrast, prefer two-sided information even under conditions of threat.

Given that political conservatives possess stronger needs for order, structure, consistency, and closure and weaker tolerance for uncertainty and ambiguity [21], it is plausible that they would be more strongly motivated to avoid the arousal of cognitive dissonance (and perhaps even the *potential* for dissonance arousal), in comparison with liberals. Consistent with this notion, a few studies indicate that selective exposure is more prevalent on the political right than the left [11], [13], [14]. For instance, Iyengar et al. [15] monitored the “clicking” habits of computer users during the 2000 U.S. presidential campaign and discovered that conservatives accessed information about Republican candidate George W. Bush significantly more often than information about Democratic candidate Al Gore, whereas liberals chose to read information about Bush and Gore more or less equally. Work on selective exposure suggests that conservatives may avoid attitude-inconsistent information more than liberals, but to our knowledge the possibility that there are ideological differences in dissonance avoidance more generally has never been tested directly.

### The Current Research

People do not experience cognitive dissonance when they are *compelled* by overwhelming force of circumstance to think or act in a way that is contrary to their own beliefs. It would appear that dissonance arousal requires some degree of choice or volition [37], [38], [39], so that for dissonance to arise people must feel that they are thinking or behaving hypocritically [40], that is, in a counter-attitudinal manner *of their own accord*. For this reason, we would expect that there would be no ideological differences in compliance with a request to engage in counter-attitudinal thought or behavior under conditions of low perceived choice (i.e., in the absence of dissonance arousal). However, if conservatives are more strongly motivated to avoid dissonance-arousing situations, they should be less likely than liberals to comply with a request to engage in counter-attitudinal behavior under conditions of high perceived choice (i.e., when the potential for cognitive dissonance is aroused). In two experiments we investigated this possibility, using the “classic” method of asking participants to construct counter-attitudinal arguments under conditions of high vs. low perceived choice.

We also sought to determine whether conservatives would eschew dissonance-arousing tasks in general – or only in explicitly political contexts. On one hand, chronic individual differences in cognitive and motivational styles could lead liberals and conservatives to differ in terms of dissonance avoidance even when it comes to nonpolitical topics. On the other hand, political (vs. nonpolitical) issues may be of much greater importance or commitment to most people, especially those who identify themselves as either liberal or conservative. For ideologues, political issues would likely possess greater potential for arousing dissonance, in comparison with nonpolitical issues. The discussion of explicitly political (vs. nonpolitical) issues would probably also increase the personal salience of ideological commitments, thereby exacerbating social and psychological differences between liberals and conservatives.

## Experiment 1: Bush vs. Obama

In Experiment 1, we investigated the hypothesis that political orientation would moderate responses to a dissonance-arousing situation. Specifically, we compared supporters of George W. Bush, a conservative, Republican president, to supporters of Barack Obama, a liberal, Democratic president, when both were instructed to construct counter-attitudinal essays in political and non-political domains. We hypothesized that those who were more politically conservative (i.e., those who preferred Bush over Obama) would be more motivated to avoid the dissonance-arousing political task than those who were more liberal (i.e., those who preferred Obama over Bush), especially under circumstances of high (vs. low) choice. We also examined the possibility that ideological differences would arise with respect to non-political (Mac vs. PC) as well as political preferences.

### Method

#### Ethics statement

The study was approved by the University Committee on Activities Involving Human Subjects (UCAIHS), the Institutional Review Board at New York University. All participants provided written informed consent prior to participation in the study.

#### Participants

One hundred and eighty participants (109 females; mean age  = 34) in the United States were recruited online through Amazon's Mechanical Turk between October 2011 and January 2012 (see [41] for a discussion of this platform as a research tool). They participated in a study of “Social Judgments and Decisions” that required them to “brainstorm on topics covered in the media” and were paid $0.25 USD; there was no penalty for failing to complete the study.

#### Materials and Procedure

All participants used their own computers to complete the study. We first solicited participants' attitudes concerning the two most recent U.S. presidents, George W. Bush and Barack Obama. Specifically, we asked, “Do you approve or disapprove of the way George W. Bush [Barack Obama] handled his job as president?” Responses ranged from 1 (strongly disapprove) to 9 (strongly approve). We also asked participants to indicate their attitudes toward two computer products, Macs and PCs (e.g., “Do you like or dislike using Mac [PC] computer products?”). Responses ranged from 1 (strongly dislike) to 9 (strongly like). Participants were also asked which president they preferred with a binary response option (i.e., “In your opinion, who has been the better president, George W. Bush or Barack Obama?”), and which type of computer they preferred (i.e., “In your opinion, which is a better computer product, PC or Mac?”). We used the binary outcome to determine which essay would be considered counter-attitudinal for each participant. Computer preferences (coded as 0 =  PC, 1 =  Mac) were weakly correlated with presidential preferences (0 =  Obama, 1 =  Bush), r (165)  = −.13, p = .09.

Using the classic “induced compliance” paradigm [39], [42], [43], we asked participants to write two counter-attitudinal essays, one on the subject of presidents and another on the subject of computers. To foster compliance, the instructions mentioned that “an important aspect of general intelligence is the ability to craft logical arguments arguing positions you may not personally endorse.” This wording was used to encourage participants to attempt counter-attitudinal essays even when they were explicitly given the option to decline the request. All participants were instructed to write two counter-attitudinal essays (one about politics and one about computers), and the order of the essays was counterbalanced.

We used the same instructions employed in classic studies of induced compliance [27]. Participants assigned to the *high choice* condition were told, “At the moment, we don't have enough of certain kinds of essays, and we need to collect several more. We would really, really appreciate it if you would help us out by writing one. Please, would you be willing to write an essay arguing that Barack Obama is [George W. Bush was] a better president than George W. Bush was [Barack Obama is]? Would you be willing to do this for us?” Participants assigned to the *low choice* condition were simply instructed: “You are assigned to write an essay arguing that Barack Obama is [George W. Bush was] a better president than George W. Bush was [Barack Obama is].”

Because we were interested in reactions to dissonance-arousing situations, all participants were asked to write counter-attitudinal essays. Thus, if a participant indicated in the initial survey that he or she preferred George W. Bush and Macs over Barack Obama and PCs, respectively, this participant would be instructed to write essays arguing that Obama is a better president than Bush and that PCs are better computers than Macs. Participants assigned to the *high choice* condition were able to respond “yes” or “no” to the request; if they responded “yes,” they were directed to the essay task, and if they responded “no,” they were instead taken to the next section of the experiment. Participants assigned to the *low choice* condition were simply directed to the essay-writing task.

Once they entered the essay task, participants were guided through a “brainstorming process,” with prompts such as: “Please think of a title,” “Please write the first main point of your argument,” “Please write the second main point of your argument,” and “Please state a conclusion to your argument.” At the conclusion of the experiment, participants responded to the same attitude items administered earlier, except that these were now embedded in a list that included filler items. They also provided demographic information, including their political orientation, which could range from 1 (*extremely liberal*) to 11 (*extremely conservative*).

Thirteen participants (6 from the low choice condition and 7 from the high choice condition) were excluded from the main analyses (leaving 167 participants, including 99 females) because they wrote *pro*-attitudinal essays despite having received instructions to write counter-attitudinal essays. (Results were nearly identical to those presented here when data from these participants was retained).

### Results and Discussion

To investigate our hypothesis, we conducted a binary logistic regression that tested for main and interaction effects of ideological preference (support for Bush [coded as 1] vs. Obama [−1]), perceived choice (high [1] vs. low [−1]), and essay content (political [1] vs. computer [−1]) on compliance behavior (did not comply [0] v. complied [1]). It was necessary to use logistic regression because of the categorical nature of the outcome variable (compliance). Predictor variables were effects-coded to facilitate the drawing of directional conclusions (relative to the overall mean or intercept).

Consistent with a forced choice dissonance paradigm, ideological asymmetries were assessed in terms of either/or categorical preferences for Bush vs. Obama. Unsurprisingly, categorical preferences were strongly correlated with political orientation for those who reported it, *r* (165)  = .56, *p*<.001. Those who preferred Bush over Obama (*M* = 7.06, SD  = 2.29) were indeed more conservative than those who preferred Obama over Bush (*M* = 3.91, SD  = 2.12), *t* (154)  = −8.62, *p*<.001.Furthermore, those who preferred Bush clearly approved of him (*M*  =  6.39, *SD*  = 1.73) and disapproved of Obama (*M* = 2.63, *SD*  = 1.82), *t* (50)  = 10.38, *p*<.001, whereas those who preferred Obama approved of him (*M*  = 5.60, *SD* = 1.99) and disapproved of Bush (*M* = 2.47, *SD*  = 1.64), *t* (115)  = −13.78, *p*<.001.

We used generalized estimating equations to determine the effects of ideological preferences, perceived choice, and essay content on compliance behavior. We hypothesized that conservative supporters of President Bush would be more motivated to avoid dissonance and therefore less likely to comply with the request to write a counter-attitudinal essay under conditions of high (vs. low) choice, in comparison with liberal supporters of President Obama. In fact, we found that *no* Bush supporters who were assigned to the high choice condition complied with the request to write an essay favoring Obama over Bush. Because the analysis could not be performed with an empty cell, we selected one participant at random and recoded his compliance status. This recoding entails a more stringent test of our hypothesis.

The analysis yielded a main effect of perceived choice, indicating that participants assigned to the high choice condition (*M* = .28, where 1 =  compliance by all participants) were much less likely than those assigned to the low choice condition (*M* = .89) to write a counter-attitudinal essay, *b* = −1.88, *SE*  = .25, Wald  = 56.94, *p*<.001, setting aside ideological preferences (for the time-being). (Note that all Wald statistics reported are Wald chi-square values with one degree of freedom.) A main effect of essay content revealed that participants were also less likely to comply with instructions to write a counter-attitudinal political essay (*M* = .46) than a nonpolitical essay (*M* = .59), *b* = −.66, *SE*  = .21, Wald  = 10.23, *p* = .001. A main effect of ideological preferences indicated that Bush supporters (*M* = .48) were less likely to comply than were Obama supporters (*M* = .55) in general, *b* = −.52, *SE*  = .25 Wald  = 4.29, *p* = .04. None of the two-way interactions attained conventional levels of statistical significance. The analysis did yield a significant three-way interaction involving ideological preference, choice condition, and essay content, *b  = *−.49, *SE*  = .21, Wald  = 5.67, *p* = .02.

To examine the nature of this interaction, we conducted simple slopes analyses within the overall logistic regression model, given that the outcome (compliance) was dichotomous in nature [44]. For each simple comparison in this experiment and the next, we recoded variables to reflect the relevant reference group for the specific contrast of interest. To compare the behavior of those who preferred Bush vs. Obama, we dummy-coded all of the predictor variables (ideological preferences: 0 =  Obama, 1 =  Bush; choice condition: 0 =  high choice, 1 =  low choice; essay content: 0 =  president, 1 =  computer). As hypothesized, we found that those who preferred Bush (*M* = .04) were less likely to comply with the dissonance-arousing, politically relevant task than those who preferred Obama (*M* = .28), *b = *−2.36, *SE* = 1.05, Wald  = 5.03, *p* = .03, under circumstances of high perceived choice. However, those who preferred Bush (*M* = .87) were not significantly different from those who preferred Obama (*M* = .80) under low choice with respect to the political task, *b = *.51, *SE*  = .72, Wald  = .50, *p* = .48. Nor were they less likely to comply with instructions to write a counter-attitudinal nonpolitical essay (about computers) under high choice (*M* = .25), in comparison with Obama supporters (*M* = .38), *b = *−.61, *SE*  = .50, Wald  = 1.49, *p* = .22 (see Figure 1). These results suggest that there was indeed an ideological difference in terms of compliance with a dissonance-arousing task, such that Bush supporters were much more likely to avoid the task in comparison with Obama supporters, but only under high choice and when it concerned a topic of political significance.

**Figure 1:** The percentage of Bush and Obama supporters in Experiment 1 who complied with instructions to write a counter-attitudinal essay in political and nonpolitical domains under conditions of low and high choice. *Note:* There were no compliers among Bush supporters under conditions of high choice with respect to the request to write a counter-attitudinal presidential essay. * *p*<.05, two-tailed.

We also conducted a parallel analysis in which political orientation was treated as a continuous measure of ideological preference (with the caveat that this measure was administered after the experimental manipulation, near the end of the experiment). Results were very similar to those summarized above. The analysis yielded a main effect of perceived choice, indicating that participants assigned to the high choice condition were less likely than those assigned to the low choice condition to comply with instructions to write a counter-attitudinal essay, *b* = −1.70, *SE*  = .22, Wald  = 61.37, *p*<.001. As before, there was also a main effect of essay content, such that participants were less likely to write a counter-attitudinal essay in the political than nonpolitical domain, *b* = −.57, *SE*  = .15, Wald  = 14.75, *p*<.001. A main effect of political orientation revealed that greater conservatism was associated with a decreased likelihood of compliance, *b* = −.14, *SE*  = .06, Wald  = 6.06, *p* = .01. This main effect was qualified by a pair of two-way interactions, which suggested that the relationship between conservatism and decreased compliance was stronger for (a) the nonpolitical than the political topic (*b* = .07, *SE*  = .03, Wald  = 4.36, *p* = .04), and (b) under conditions of high (vs. low) choice (*b* = −.10, *SE*  = .06, Wald  = 3.25, *p* = .07). In addition, a significant three-way interaction involving political orientation, essay content, and choice condition was observed, *b* = −.14, SE  = .03, Wald  = 18.99, *p*<.001. Simple slopes analyses revealed that, consistent with predictions (and the results summarized above), greater conservatism was associated with a decreased likelihood of complying with instructions to write a counter-attitudinal political essay under circumstances of high perceived choice (*b* = −.31, *SE* = .10, Wald  = 10.54, *p* = .001). This pattern did not emerge with respect to the political task under low choice conditions; in fact, there was a marginal tendency for conservatives to comply slightly more often with instructions, *b* = .18, *SE*  = .10, Wald  = 3.28, *p* = .07. There was an even weaker relationship between political orientation and likelihood of compliance with instructions to write a counter-attitudinal essay on a nonpolitical topic (computer preferences) under conditions of high choice, *b* = −.17, SE  = .10, Wald  = 2.75, *p* = .10.

## Experiment 2: Reagan vs. Clinton

The purpose of Experiment 2 was to replicate and extend the findings of Experiment 1. There are a number of factors in addition to political ideology that might have contributed to the difference in compliance behavior we observed with respect to Bush and Obama supporters. For instance, the fact that Obama was the current President (and would be seeking re-election) may have increased resistance among his ideological adversaries (who were in the midst of selecting his Republican opponent during the time of data collection). Conversely, Obama supporters may have been more willing to argue in favor of Bush because he was no longer running the country, or because of strong national support for him in the aftermath of the terrorist attacks of September 11, 2001. Therefore, we conducted an additional experiment with a different pair of presidents, namely Ronald Reagan and Bill Clinton. These are both former two-term presidents who do not differ in terms of race (as Bush and Obama do) and who left office with similar public approval ratings [45]. Following the results of Experiment 1, we made the strong directional prediction that those who preferred Reagan would be less likely to comply with a dissonance-arousing political task (under high choice) in comparison with those who preferred Clinton.

### Method

#### Participants

One hundred fifty-nine participants (90 females, 2 declined to indicate sex; mean age  = 33) in the U.S. were recruited online through Amazon's Mechanical Turk from November 2011 to January 2012. Nine participants (3 from the low choice condition and 6 from the high choice condition) were excluded from the main analyses (leaving 150 participants, including 86 females) because they wrote pro-attitudinal essays despite having received instructions to write counter-attitudinal essays. (Results were nearly identical to those presented here when data from these participants was retained.)

#### Materials and Procedure

The general procedure was identical to that of Experiment 1, except that participants were asked to write counter-attitudinal essays on two new topics: (a) whether Bill Clinton or Ronald Reagan was the better president, and (b) whether coffee or tea is the superior drink. Consistent with the results of pilot testing, study participants' beverage preferences (coded 0 =  coffee, 1 =  tea) were uncorrelated with their political preferences (coded 0 =  Clinton, 1 =  Reagan), r (148)  = .002, p = 98.

### Results and Discussion

To assess our predictions, we conducted a binary logistic regression that tested for main and interaction effects of ideological preference (support for Reagan [coded as 1] vs. Clinton [−1]), perceived choice (high [1] vs. low [−1]), and essay content (political [1] vs. beverage [−1]) on compliance behavior (did not comply [0] v. complied [1]). As in Experiment 1, presidential preferences were significantly correlated with general political orientation, *r* (148)  = .43, *p*<.001. Those who preferred Reagan over Clinton (*M* = 6.89, *SD*  = 2.81) were indeed more conservative than those who preferred Clinton over Reagan (*M* = 4.53, *SD*  = 2.12), *t* (148)  = −5.80, *p*<.001. Furthermore, those who preferred Reagan approved of him (*M* = 7.17, *SD*  = 1.82) more strongly than they approved of Clinton (*M* = 4.70, *SD*  = 2.10), *t* (53)  = 7.42, *p*<.001, and those who preferred Clinton approved of him (*M* = 6.88, *SD*  = 1.60) more than they approved of Reagan (*M* = 4.49, *SD*  = 1.60), *t* (95)  = −11.44, *p*<.001.

We again used generalized estimating equations to determine the effects of ideological preferences, perceived choice, and essay content on compliance behavior. Because we had a strong prediction that those who preferred Reagan would comply less than those who preferred Clinton, we used one-tailed tests to assess simple contrasts but report the results of both one-tailed and two-tailed tests for the sake of clarity and completeness. The analysis yielded a main effect of choice condition, indicating that participants under high perceived choice (*M* = .25) were much less likely than those under low choice (*M* = .88) to agree to write a counter-attitudinal essay, *b* = −1.67, *SE*  = .21, Wald  = 63.68, *p*<.001. A main effect of essay content revealed that participants were less likely to comply with the task when it involved politics (*M* = .45), as compared with beverages (*M* = .58), *b* = −.52, *SE*  = .16, Wald  = 10.02, *p* = .002. No other main or interaction effects attained conventional levels of significance.

To probe our focal hypothesis that those who preferred Reagan would be less likely than those who preferred Clinton to comply with a dissonance-arousing task in the political domain, we again conducted simple slopes analyses to spotlight the specific comparisons of interest [44]. We dummy-coded the predictor variables as follows: ideological preference: 0 =  Clinton, 1 =  Reagan; choice condition: 0 =  high choice, 1 =  low choice; essay content: 0 =  president, 1 =  beverage. Consistent with our directional hypothesis (See Figure 2), under high choice Reagan supporters (*M* = .10) were less likely to comply with the request to write a counter-attitudinal political essay than were Clinton supporters (*M* = .22), *b = *−1.36, *SE*  = .80, Wald  = 2.91, *p* = .044, one-tailed (*p* = .088, two-tailed). Under low choice, no effect of ideological preference was observed *b = *−.68, *SE*  = .68, Wald  = 1.00, *p* = .16, one-tailed (*p* = .32, two-tailed). Those who preferred Reagan (*M* = .79) were as likely as those who preferred Clinton (*M* = .84) to write a counter-attitudinal essay about politics under conditions of low choice. No differences were observed either between those who preferred Reagan (*M* = .30) and Clinton (*M* = .38) in terms of compliance with instructions to write a counter-attitudinal essay about coffee vs. tea under high choice, *b = *−.42, *SE*  = .50, Wald  = .71, *p* = .20, one-tailed (*p* = .40, two-tailed). Replicating Experiment 1, these results lend further support to the notion that there is an ideological difference in reactions to dissonance-arousing situations, insofar as those who preferred Reagan (vs. Clinton) were more likely to avoid a highly dissonant task–but only when it involved a political topic.

**Figure 2:** The percentage of Reagan and Clinton supporters in Experiment 2 who complied with instructions to write a counter-attitudinal essay in political and nonpolitical domains under conditions of low and high choice. * *p*<.05, one-tailed; *p*<.10, two-tailed.

Once again, we conducted a parallel analysis in which political orientation was treated as a continuous measure of ideological preference, despite the fact that this measure was taken at the end of the experiment, following the experimental manipulation. This analysis yielded a main effect of choice, such that participants assigned to the high choice condition were less likely than those assigned to the low choice condition to write a counter-attitudinal essay, *b* = −1.61, *SE*  = .20, Wald  = 63.58, *p*<.001. A main effect of essay content revealed that compliance was lower in the political than nonpolitical domain (overall), *b* = −.41, *SE*  = .15, Wald  = 7.34, *p* = .007. No other main or interaction effects reached conventional levels of significance. Simple slopes analyses failed to identify significant effects of political orientation on compliance with instructions to write a counter-attitudinal political essay under conditions of high (*b* = −.01, *SE* = .11, Wald  = .004, *p* = .95) or low choice (*b* = −.21, *SE* = .15, Wald  = 2.02, *p* = .16). Political orientation was also unrelated to compliance with instructions to write a counter-attitudinal essay in a nonpolitical domain under high choice, *b* = .02, *SE* = .09, Wald = .04, *p* = .85. Thus, the results of Experiment 2 replicated those of Experiment 1 when ideological preferences were estimated using categorical (either/or) presidential preferences but not when they were estimated using the continuous measure of political orientation administered at the end of the experiment. We will return to this issue in the General Discussion.

## General Discussion

The current research suggests that, in some situations at least, conservatives avoid dissonance-arousing situations to a greater extent than liberals do. Specifically, we found that supporters of Republican presidents were less likely than supporters of Democratic presidents to comply with instructions to write counter-attitudinal essays under circumstances of high perceived choice. This result was specific to the political domain. That is, the ideological difference was observed when participants were asked to write an essay in favor of their less preferred president but not when they were asked to write an essay in favor of their less preferred computer brand or beverage. These results suggest that there are ideological differences in the avoidance of situations that have the potential to arouse cognitive dissonance.

One of the most striking results is that we could not find a *single* Bush supporter who was willing, when given a choice, to write a counter-attitudinal essay suggesting that Obama is a better president than Bush was. Some conservatives found the task instructions themselves to be extremely distasteful, making post-study comments such as: “Yeah who would actually aprove [*sic*] of the job Obama has done? I mean really!” and “Not for all the tea in China would I write that.” Similar patterns were observed with respect to Reagan and Clinton supporters, but the ideological difference was weaker, possibly because both presidents left office with high job approval ratings and are now considered to be among the two best presidents in recent history [46], which may render them easier (and therefore less dissonance-arousing) to praise.

To be sure, neither liberals nor conservatives were enthusiastic about writing a counter-attitudinal political essay, but several Obama supporters did undertake the dissonance-arousing task under high choice, writing statements such as: “George Bush did what he said he was going to do but Obama filled us with liberal false promises,” and “There were extended periods of economic growth under George W. Bush, while the economy has lagged badly under Barack Obama.” Given an opportunity to provide post-study feedback, one Obama supporter said that she “hated having to brainstorm in support of Bush” but still managed to write a counter-attitudinal essay under high perceived choice. Another liberal apparently enjoyed the exercise, commenting, “This was fun!” In contrast, no Bush supporters agreed to write pro-Obama essays under high choice, nor did any of them state that the exercise was “fun.” The ideological difference we observed appears to be a *relative* (rather than an absolute) difference in dissonance avoidance.

Our findings are broadly consistent with previous work on selective exposure. Many studies have shown that individuals avoid exposure to potentially dissonance-arousing, attitude-incongruent information, especially when such information is high in personal or ideological relevance [7], [29], [30], [47]. Insofar as many people hold stronger attitudes about political than non-political matters (such as computer brands and beverages), it may not be too surprising that dissonance avoidance would be more common in the political domain. Our work suggests that this is the case, although it may be that the non-political preferences we focused on were too weak to arouse dissonance. Thus, future work may reveal that liberal-conservative differences in dissonance avoidance do emerge with respect to non-political tasks as long as the topic is of genuine importance to research participants.

An alternative explanation for the ideological discrepancy in compliance behavior is that conservatives were more sensitive than liberals to cues communicating descriptive social norms. It is conceivable, for instance, that the wording of the instructions in the high choice condition, which suggested that there was a shortage of certain kinds of essays, was interpreted as indicating that very few people were willing or able to argue in favor of President Obama or Clinton. There is indeed evidence that conservatives value conformity more than liberals do [48], [49] and possess stronger desires to “see the world as others who share their beliefs generally do” [Stern, West, Jost, & Rule, unpublished data]. Perhaps conservatives took the experimental request as encouragement to join others in *not* writing an essay supporting a liberal president. Alternatively, liberals may have been more motivated than conservatives to test their “ability to craft logical arguments.” Importantly, however, we observed no ideological differences in willingness to comply with the same instructions when participants were asked to write counter-attitudinal essays on non-political topics.

In both experiments, we supplemented our primary statistical analyses, which operationalized ideological preferences in terms of categorical (either/or) preferences for one president over another, with additional analyses using a continuous measure of political orientation (administered at the end of the experimental sessions). With respect to Experiment 1, the results were virtually identical for the two types of analyses. For Experiment 2, however, the hypothesized pattern emerged when ideological preferences were treated as a categorical variable but not as a continuous measure. It is possible that this difference is attributable to the fact that, as cognitive dissonance theorists have argued, the act of *choosing* one stimulus over another is critical to the experience of dissonance arousal [37]. Indeed, this is why we employed a “forced choice” paradigm (which excludes middle-of-the-road responding) in the present research program. Another possibility is that, psychologically speaking, slight liberals may have more in common with moderate and extreme liberals than with slight conservatives (and vice versa). This would also produce nonlinear rather than linear effects of ideological preferences. In any case, future research would do well to address this possibility in a systematic manner.

Our finding that political conservatives were less willing than liberals to engage in dissonance-arousing tasks is in line with previous theory and evidence concerning ideological differences in cognitive and motivational styles [20], [21]. Our work may also help to explain serendipitous results from other research programs. For example, Iyengar et al. [15] observed that conservative voters were less likely than liberal voters to expose themselves to information about their non-preferred presidential candidate during the election of 2000. In addition, MacCoun and Paletz [50] found that conservatives were more likely than liberals to dismiss as inherently biased research that supports politically unwelcome conclusions (e.g., that the death penalty fails to deter criminals). It is quite possible that ideological differences in dissonance avoidance account for these asymmetries in behavior and judgment, and they may also suggest circumstances under which conservatives might be more strongly committed to partisan causes, in comparison with liberals (see also [51]).

If there are indeed ideological differences in the tendency to avoid dissonance-arousing thoughts, as our data suggest, this may also help to explain why conservatives are more prone to engage in biased forms of moral reasoning [12] and more likely to hold false beliefs concerning a number of public policy issues [52], in comparison with liberals. Nyhan and Reifler [16] observed how liberals and conservatives would respond to the presentation of evidence contradicting their prior (incorrect) beliefs. They found that conservatives exhibited a “backfire effect,” reporting even *stronger* commitment to their initial beliefs after being exposed to discrediting evidence. Liberals failed to correct their initial misperceptions in the face of disconfirming information, but they did not exhibit a backfire effect.

Cooper and Mackie [53] found that when members of a Ronald Reagan election group were asked to come up with (attitude incongruent) statements in favor of President Jimmy Carter during the campaign of 1980, they resolved their dissonance by derogating Democrats rather than changing their initial attitudes toward Reagan's election. However, when Reagan supporters were asked to come up with counter-attitudinal statements on a topic that was related but tangential to the group's purpose, they exhibited classic cognitive dissonance effects, including attitude change. Because Carter supporters were not examined in Cooper and Mackie's research, it is unclear whether this result was specific to conservatives or more generally applicable. In future work it would be useful to investigate the possibility that, following compliance with a dissonance-arousing political task, conservatives bolster their initial attitudes and derogate their ideological opponents more than liberals do.

It should be noted, at least in passing, that epistemic disadvantages (such as attitude bolstering and avoidance of disconfirming information) might translate into real political advantages (such as commitment and loyalty) when it comes to the ballot box. At the same time, the refusal to consider opposing points of view in good faith may hinder the functioning of a democratic society [2]. An unwillingness to consider or express attitude incongruent information may be related to a lower capacity for perspective-taking, which has been linked to stereotyping and intergroup bias [54]. These outcomes, too, could affect the nature of political discourse in a pluralistic society. To the extent that the avoidance of dissonance-arousing situations exacerbates political gridlock and ideological polarization, a detailed scientific understanding of the role of ideology in motivating dissonance avoidance is sorely needed. It may even inspire the design of novel communication strategies that will help to overcome ideological divides that otherwise seem unbridgeable.
